RETRACTED

# Current Status of Malignant Tumors after Organ Transplantation

**DOI:** 10.1155/2022/5852451

**Published:** 2022-02-18

**Authors:** Bairu Shen, Zhuofei Cen, Minghua Tan, Changshan Song, Xuhui Wu, Jiaqing Wang, Minqian Huang

**Affiliations:** Thoracic Surgery, Foshan Clinical Medical School of Guangzhou University of Chinese Medicine, Guangdong Province, China

## Abstract

**Objective:**

To analyze the diagnosis and treatment of patients with concomitant malignant tumors after organ transplantation by compiling data from organ transplantation patients.

**Methods:**

By searching CNKI and PubMed databases, we made a systematic analysis of the studies of postorgan transplantation complicating malignant tumors in the last decade.

**Results:**

There were 10 articles on malignant tumors after renal transplantation, 8 articles on liver transplantation, 2 articles on heart transplantation, and 1 article on lung transplantation. The incidence of malignant tumors complicating renal transplantation is 10.4% in Europe, with skin cancer and Kaposi's sarcoma being common; the incidence in the United States is 3.4%, with PTLD having the highest incidence; the incidence of malignant tumors is relatively lowest in Asia, with gastrointestinal malignancies being the main ones. The mean time to complication of malignancy after renal transplantation is 3.83 years. The incidence of concurrent malignancies after liver transplantation is 8.8% in Europe, where skin cancer and Kaposi's sarcoma are common; 5.6% in Asia, where gastrointestinal tract tumors are prevalent; and 4.5% in the United States, where gastrointestinal tract tumors, PTLD, and hematologic diseases are predominant. The mean time to complication of malignancy after liver transplantation is 4.79 years. The incidence of malignancy after heart transplantation is 6.8-10.7%. The incidence of malignancy after lung transplantation is about 10.1%. Minimization of immunosuppression or modification of immunosuppression regimens may be a key component of cancer prevention. mTOR inhibitors and phenolate (MMF) reduce the incidence of de novo malignancies in patients after solid organ transplantation. Surgical treatment improves survival in patients with early malignancies. The use of external beam radiation therapy in the treatment of hepatocellular carcinoma is limited due to the risk of radiation liver disease.

**Conclusions:**

The risk of concomitant malignancy needs to be guarded for 5 years of immunosuppressive therapy after organ transplantation surgery. Adjusting the immunosuppressive treatment regimen is an effective way to reduce concurrent malignancies. Systemic chemotherapy or radiotherapy requires vigilance against the toxic effects of drug metabolism kinetics on the transplanted organ.

RETRACTED

## 1. Introduction

In recent years, with the advance of surgical technology and the application of immunosuppression, transplantation has merged as the best treatment for end-stage carcinoma of solid organs, which extended graft and patient survival after transplant. However, the morbidity and mortality rates of patients with recurrent malignancies after organ transplantation had increased [1]. Compared with the general population, patients with organ transplant have a higher risk of developing carcinoma by 2.6 times [2]. Over the years, tumors have become an important cause of death among solid organ transplant recipients, and it is foreseen that it would take the first place of cardiovascular disease in mortality within the next 10 years [3, 4]. Some malignant tumors are caused by the oncogenic viruses leading to the loss of immune control, while others are not related to known infections [5]. The possible occurrence mechanism is that under medicine-induced low immune surveillance, the virus disrupts the differentiation of infected cells by disrupting cell cycle control [6]. Other causes of certain cancers may include chronic immune disorders or inflammation, potential medical conditions, or other factors such as drug toxicity. Immunosuppression has undoubtedly raised the positive outcomes in recipients after organ transplant but also increased the risk of infection. Patients are also relatively less tolerant of cancer treatment. A systematic literature examination about the morbidity and the treatment of de novo malignancies (DNM) after different solid organ transplantation was described. Worldwide data were collected from related articles in PubMed and CNKI. Data from various experiences were reported and compared to access a clear clinical guideline.

## 2. Material and Methods

### 2.1. Search Strategy

A literature review was conducted in March 2021 through PubMed and CNKI databases to find studies pertaining to organ transplantation, malignant tumor, immunosuppression, and chemical therapy threshold. Articles published in languages other than Chinese and English were excluded. The publishing year is between 2011 and 2021. All texts were full text accessible. The keywords are (de novo malignancies after organ transplantation) AND (treatment).

### 2.2. Inclusion and Exclusion Criteria

Articles published in journals describing the morbidity of the malignant tumor after solid organ transplantation and its treatment were searched. Data from kidney, gastrointestinal, lung, posttransplant lymphoproliferative diseases (PTLD), and other DNM were collected and discussed from systematic reviews, randomized clinical trials, observational studies, and case-control studies. 10-year limits were applied to access the up-to-date treatments in this field. Non-English articles in PubMed and articles with no specific number of patients and the number of patients with tumors were excluded from this review. A total of 10 articles on malignant tumor after kidney transplantation, 8 articles on liver transplantation, 2 articles on heart transplantation, and 1 article on lung transplantation were screened out.

RETRACTED

### 2.3. Research Method

The incidence of malignant tumors after organ transplantation and the types of malignant tumors with the highest incidence were analyzed. The types of tumors susceptible to different regions were analyzed, and the current diagnosis and treatment after various organ transplantation were summarized.

## 3. Results

### 3.1. Incidence of Concurrent Malignancies after Kidney Transplantation

Ten articles (Table 1) reported the morbidity of malignant tumors after renal transplantation in seven countries from 1966 to 2016. The incidence of posttransplant carcinoma is shown in Figure 1. Among the seven articles, Tsai et al. [7] from Taiwan, China, have reported the highest morbidity which is up to 18.8%, among which the incidence of urinary system tumor was the highest, reaching 54.3%, followed by the case data reported by Apel et al. [8] from Germany, of which the incidence of tumor was 12.3%, among which the incidence of gastrointestinal tumor was the highest, reaching 18.6%. Fröhlich et al. [9] reported that the incidence of tumor was 10.7% in the study of the UK, and the incidence of renal cancer was the highest among the reported cases, which was 31.8%. The article did not include patients with nonmelanic skin cancer. Mazzucotelli et al. [10] reported that the incidence of malignant tumors in kidney transplant patients in Italy was 10.2%, among which PTLD had the highest morbidity which is 34.7%. In the article reported by Zavos et al. [11] from Turkey, the incidence of tumor was 9.7%, and the highest incidence is 49.7% of skin cancer. The Italian data reported by Rossetto et al. [12] have shown the incidence of posttransplant tumor was 9.3%, and the highest morbidity was 28.8%, which is gastrointestinal tumor. Gioco et al. [13] reported that the incidence of tumors from Italy was 7.3%, and the highest incidence of skin cancer was 23.7%. Sampaio et al. [14] from the United States have reported that the incidence of posttransplant tumor was 3.4%, and the morbidity of PTLD was the highest which was 21.3%. Park et al. [15] from South Korea reported that the incidence of tumor was 2.7%, and the incidence of gastrointestinal tumor was the highest which is 34.6%. Wu et al. [16] reported that the incidence of tumor in China was 0.95%, among which the incidence of the urinary system was the highest, reaching 50%.

RETRACTED

It can be seen that tumor viruses are prone to invade different organs among kidney transplant patients in different countries and regions and the data from different centers were quite different. Among the data reported by three centers in Italy, the highest morbidity of tumor was, respectively, skin cancer, lymphatic system, and gastrointestinal carcinoma.

Generally speaking, Europe has a higher incidence of skin cancer, which is 23.7%-49.7% in Turkey and Italy. Lymphoid tumors and gastrointestinal tumors have the morbidity of 21.3%-34.6% in North America and South Korea, and 50% of the posttransplant carcinoma in China is urinary tumor. The statistical results in our review are in conformity with domestic literature reports, the incidence of skin cancer and the proportion of which were significantly lower than the European and American countries; this may be related to skin color, the sunshine radiation, and the discrepancy in the demand of immunosuppression [17]. In China, the high risk of urology malignant tumor after renal transplantation may be due to our race, the discrepancy in type, and dosage of immunosuppression. The following reason was that when the transplanted kidney starts to work, the original kidney will not secrete urine or reduce urine secretion, which weakens the flushing effect on the urinary tract and keeps the metabolites in the urinary tract, thus continuously stimulating the urethral epithelial cells and eventually leading to renal tumor [18].

In summary, we have summarized the data on tumors after renal transplantation according to regions. The incidence of tumors after renal transplantation in Europe amounted to 10.4%, with skin cancer and Kaposi's sarcoma, and the highest incidence of gastrointestinal cancers, accounting for 16.2% of all patients with cancer. Only one country in North America has data from the United States, whose tumor incidence rate is 3.4%, with PTLD having the highest incidence rate of 21.3%. Asia has the relatively lowest tumor incidence rate of 2.9%, with the incidence of gastrointestinal tumors reaching 33.2%.

This shows that the prevalence of tumors that tend to complicate kidney transplant patients in different regions is inconsistent, with a higher incidence of skin cancer in Europe, which may be related to differences in skin color, sun exposure to radiation, and the need for immunosuppressive agents [17]. Although the incidence of gastrointestinal tumors is higher in Asia, the reason for this may be related to Asian dietary habits. However, in the Korean data by Park et al. [15], it was shown that non-Hodgkin's lymphoma, Kaposi's sarcoma, skin cancer, and leukemia (in men) were higher after transplantation compared to the general population in terms of the standardized incidence of cancer than SIR. This is similar to data from the United States, where the high prevalence of lymphatic system neoplastic disease may be related to a more sensitive lymphatic system to immunosuppression, which may lead to a higher proliferation of EBV.

RETRACTED

### 3.2. Morbidity of Carcinoma of Postliver Transplantation

It is summarized in Table 2 the data of malignant tumor after liver transplantation in eight centers in 1988-2017 years. The epidemiological data is detailed in Figure 2. We can conclude that the incidence of tumors in France and Germany is relatively high, reaching 16.5%~22.8%, followed by Japan, 11.4%, and the morbidity of tumor in Italy and Korea is 5.6% and 5.5%, respectively. The morbidity of cancer in Saudi Arabia is 3.4%, and the lowest ones are 2.2% and 0.2% reported by two Turkey centers. Specific data is shown in Figure 2. Among the cases in France and Germany, the incidence of skin cancer was the highest, reaching 29.2%~31.2%. In South Korea, the morbidity of gastrointestinal tumors was 46.9%, and the incidence of PTLD in Saudi Arabia was higher than that in Turkey, reaching 62.5%~63.1%. The incidences of gastrointestinal tumors and PTLD are both high in Japan. Youn et al. [19] concluded that colorectal malignancies are dominant in Japanese liver transplant recipients. It was consistent with the results concluded in our review.

In summary, we conclude that the incidence of postliver transplantation tumors is higher in Europe at 8.8%, with skin cancer and Kaposi's sarcoma accounting for 20.9% of all tumors and PTLD and hematologic tumors accounting for 20.7%. The incidence of new tumors in Asia is 5.6%, with a high incidence of gastrointestinal tumors, whose incidence is 44.4%. In North America, we take the United States as an example, where the incidence of tumors after transplantation is 4.5%, with 23.8% of gastrointestinal tract tumors and 23.7% of PTLD and hematologic disorders. This is basically consistent with the data after renal transplantation. In Europe, the incidence of skin cancer is higher, the reason of which should be related to the geographical area, while the incidence of hematologic malignancies is higher, the reason of which may be related to the use of immunosuppressive drugs. Asia has the highest incidence of gastrointestinal tumors. North America has a higher incidence of PTLD and hematologic disorders, whose only independent risk factor that can be recognized is age, while patients with liver transplantation due to HCV also have a higher risk of developing hematologic tumors [24].

RETRACTED

### 3.3. Morbidity of Carcinoma of Postheart Transplantation

Youn et al. [19] analyzed 17587 patients in the International Society for Heart and Lung Transplantation (ISHLT) from January 2000 to December 2011. It was concluded that the risk of solid malignancy from the first year to the fifth year after transplantation was 10.7%. The cumulative incidence is as follows: skin cancer (7.0%), nonskin solid cancer (4.0%), and lymphoproliferative diseases (0.9%). In the United States, about 20% of heart transplant recipients will develop skin cancer within 10 years after transplantation. In all types of cancer, the survival rate of patients with new malignant tumors was significantly lower than that of patients without malignant tumors. Meiser et al. [27] reported that seven of 103 patients who received heart transplantation from April 1999 to April 2017 were suffering from malignant tumors, which morbidity is 6.8%. Among all, 3 cases were PTLD, 1 case was squamous cell carcinoma of the skin, 2 cases had colon cancer, and 1 case had bladder cancer.

### 3.4. Morbidity of Carcinoma of Postheart Transplantation

There are few articles related to lung transplantation, and only one of which meets our screening conditions was selected whose title is “De Novo Malignancy after Lung Transplantation in Japan” [28]. It summarizes 179 lung transplantation operations performed in 7 institutions in Japan from 2001 to 2010, of which 18 recipients (10.1%) developed new malignancies. The higher incidence of malignancies was lymphoproliferative malignancies (12 cases, 1 of which were double neoplastic cancer after tongue cancer), followed by cervical cancer (4 cases), breast cancer (2 cases), and tongue cancer (1 case).

### 3.5. Immunosuppressive Therapy Analysis

The use of immunosuppression has always been heated discussed in patients after organ transplantation. Rousseau et al. [29] stated that no matter what immunosuppression regimen is adopted, posttransplant patients can benefit from the best tumor treatment, reducing the risk of death by 55%, which is acceptably safe. The article on head and neck cancer after liver transplantation reported by Graham et al. [30] also points out that induced immunosuppression does not increase the risk of carcinoma. However, in the article on concurrent tumors after liver transplantation, it is generally agreed that the minimization of calcineurin inhibitor (CNI) and the use of mTOR inhibitors can reduce the probability of recurrence or de novo tumors of hepatocellular carcinoma [31, 32].

RETRACTED

After organ transplantation, patients will generally undergo a standardized three-drug immunosuppression regimen. In the cases of urinary system diseases reported by Karczewski et al. [33], three immunosuppressive methods were selected: tacrolimus+mycophenolate mofetil+prednisolone, cyclosporin+imidazolium thiopurine+prednisolone, and cyclosporin+mycophenolate mofetil+prednisolone.

CNI is a common immunosuppressant for immunosuppression after liver transplantation. Tacrolimus (TAC) is commonly used compared with cyclosporine because it reduces the rate of acute rejection and improves the survival of both grafts and patients [34]. However, CNI has the risk of carcinogenesis, which may be related to its mechanism of inhibiting DNA repair and apoptosis. Studies have shown that cyclosporine can accelerate tumor progression through its direct effect on cells, which especially may increase the incidence of skin cancer after transplantation [35]. It has also been reported that tacrolimus may increase the incidence of tumors in vivo after transplantation [36]. While there is still a critical controversy about the side effects of CNIs, there are increasing scholars stating not using CNI immunosuppressants. Meiser et al. [27] reported that it is possible to take no CNI immunosuppressants after heart transplantation. On the one hand, it is conducive to the survival of patients, inhibits malignant tumors, protects renal function, and resists cytomegalovirus infection and vascular diseases. On the other hand, while no CNI immunosuppression after heart transplantation (HTx) has a poor effect in preventing acute rejection, the side effects are low. In the preliminary study of malignant tumors after renal transplantation, it is also proposed that the combined blocking of belatacept and mTOR inhibitors can achieve the same therapeutic effect as the standard treatment without CNI inhibitors and steroids after renal transplantation [37]. However, in Guethoff et al.'s report [38], it is pointed out that the reduction of CNIs does not lead to superior long-term renal function. Minimization or modification of immunosuppression may be a key component of cancer prevention, because the effect of immunosuppression on carcinogenesis seems to be dose-dependent. However, the risk of rejection and the benefits of cancer prevention need to be carefully weighed. In liver transplantation, the minimization of CNIs and the use of mTOR are associated with a significant reduction in the recurrence rate of hepatocellular carcinoma [39, 40]. There is no clear regulation on the amount of immunosuppressant. In Zhanwen's report on tumor after kidney transplantation [41], it is mentioned to reduce the dose of immunosuppressant to 1/2~2/3 of the original dose, and in Hao's study [42], it is mentioned to reduce the dose of immunosuppressant to 1/4~1/2.

RETRACTED

### 3.6. Antitumor Therapy Analysis

The mammalian target of rapamycin is a serine/threonine kinase involved in cell growth, proliferation, metabolism, and angiogenesis. The mTOR pathway is upregulated in many malignant tumors, so mTOR inhibition may have chemopreventive function [43]. In the liver transplant population, a retrospective study of patients with alcoholic cirrhosis liver transplant determined that conversion to everolimus-based immunosuppression can reduce the risk of noncutaneous neomalignant tumors [44]. Rapamycin has also a good therapeutic effect on Kaposi's sarcoma [45]. In the case of Kaposi's sarcoma reported by Roy et al. [46], it is pointed out that mTOR inhibition is considered to be effective in the treatment of Kaposi's sarcoma because it inhibits angiogenesis by reducing the secretion of vascular endothelial growth factor and inhibiting the formation of tumor blood vessels.

Sirolimus and everolimus are mammalian target inhibitors of rapamycin (mTOR), which have potential antiproliferative properties and are considered to inhibit tumor growth. However, the article on their antitumor effects is not systematic [47]. More and more evidence has shown that with the introduction of mTOR inhibitors, patients with gradually reduced CNI have a lower incidence of tumor diseases than subjects treated with standard dose CNI [48]. In addition, the introduction of mTOR inhibitors can reduce the risk of death in patients with de novo malignancies by 76% [30]. In addition, early use of everolimus can improve renal function which is a feasible choice for renal insufficiency after liver transplantation [49, 50].

Mycophenolate mofetil (MMF) is an antibiotic. As an antitumor drug for leukemia, lymphoma, and various solid tumors, it has an impact on tumor adhesion, angiogenesis, and EBV-infected cells, which reduce the incidence of new malignant tumors and long cancer-free survival after solid organ transplantation [51, 52]. MMF is commonly used along with TAC and steroids [53].

Anti-CTLA-4 and anti-PD1/PDL1 therapy can be used to treat recurrent or refractory classical Hodgkin lymphoma, metastatic melanoma, and other tumors by mobilizing the function of the autoimmune system and fighting against cancer cells [54, 55], bringing hope to patients with advanced tumors. However, in the vast majority of immunotherapy clinical trials, patients with organ transplantation complicating malignancies have not been studied because they may increase the risk of transplant organ rejection [56]. PD-1 and CTLA-4 channels are important processes in immune tolerance of transplanted organs, and alterations in these channels may lead to rejection of the transplanted organ by the recipient. The incidence of irAEs with anti-PD-1 drugs is much smaller than with anti-CTLA-4, so it has been hypothesized that anti-PD-1 drugs would be safer to use in organ transplant recipients, but this clearly does not correspond to our real-world data [57]. Blockade of the PD-1 pathway may lead to increased organ transplant rejection compared to CTLA-4 blockade, and the PD-1 pathway plays a more dominant role in allograft immune tolerance than the CTLA-4 pathway. [58]. Blazar et al. found that anti-PD-1 antibodies have a higher risk of causing graft-versus-host disease than anti-CTLA-4 and that the combination leads to more severe graft-versus-host disease [59]. None of the patients who develop graft rejection can be salvaged by immunosuppression [58], and the graft loss rate is as high as 80% [56]. However, some patients have responded or stabilized after immunotherapy [56]. Most scholars believe that there is no direct correlation between the risk of graft rejection and the time after organ transplantation [56], and we have not found that patients with long-term transplants are not prone to rejection when receiving immunotherapy [57]. However, people may be more reluctant to introduce immune checkpoint inhibitor therapy in the initial posttransplant period [60]. The rejection rate of allografts is relatively high in the early stages of the use of immunotherapy and is often accompanied by a high mortality rate [57].

RETRACTED

Targeted therapy in driver gene-positive malignancies, particularly in patients with non-small-cell lung cancer, is currently an effective treatment modality and has shown relatively good therapeutic effects in nonorgan transplant patients. However, data on targeted therapy for organ transplantation-complicated malignancies are less available and are dominated by scattered case reports. De Pas et al. found that the use of cyclosporine was not a contraindication to treatment with erlotinib, with no associated toxicity [61]. Hecimovic et al. reported the treatment of a patient with non-small-cell lung cancer (EGFRL585R+) complicated by heart transplantation, who was treated with cyclosporine combined with erlotinib resulted in a very good treatment of the malignancy with no significant toxic side effects or rejection of the transplanted organ [62]. However, close monitoring of drug concentrations in the blood is necessary.

### 3.7. Surgical Treatment

After kidney transplantation, surgery will be the main treatment, before the cancer has spread. Radical tumor resection can reduce the recurrence of cancer and improve the survival rate of patients. Among the cases of urinary diseases reported by McAlister et al. [34], 13 patients with renal cancer chose nephrectomy, of which 12 survived and 1 died. Cornelis et al. [63] reported that subcutaneous radiofrequency ablation is effective for renal cell carcinoma less than 4 cm. The article reported by Kluijfhout et al. [64] pointed out that the treatment of thyroid cancer after solid organ transplantation should be similar to that of thyroid cancer patients in the general population.

RETRACTED

Cheung et al. [65] reported the diagnosis and treatment of hepatocellular carcinoma after renal transplantation. All 15 asymptomatic patients received treatment, including 8 cases of hepatectomy, 2 cases of transcatheter arterial chemical embolization (TACE), 2 cases of radiofrequency ablation (RFA), 1 case of percutaneous ethanol injection (PEI), 1 case of operation+TACE, and 1 case of RFA+TACE. Nine of them survived, but one developed renal rejection. On the other hand, none of the 3 patients diagnosed by symptoms underwent surgery. One of them received selective internal radiation (SIT) and died 16 months later. The other 2 cases received symptomatic treatment and died only 1 month and 5 months after diagnosis. Therefore, surgical treatment can improve the survival rate of patients to a certain extent, but it is also related to the patient's physical state and tumor.

The same as patients with malignant tumors after renal transplantation, patients with new malignant tumors after liver transplantation can undergo surgical treatment, remove the cancerous area to prevent the spread of cancer cells, and perform lymph node dissection. Gastrointestinal tumors are common in Asia. Shimizu et al. [66] reported that gastric cancer was discovered 30 months after living donor liver transplantation. The patient underwent segmented gastrectomy and lymph node dissection. The histopathological examination of the resected stomach was pT2N1M0, phase II. Tacrolimus was stopped on the day of operation and recovered one day later. The patient did not receive chemotherapy after operation. He is still alive after more than four years. In the case of gastric cancer after liver transplantation for liver cancer reported by Yang et al. [67], the patient was successfully treated by radical distal gastrectomy and D2 lymph node dissection and was diagnosed as stage IIIC gastric adenocarcinoma (pT4aN3bM0) by pathological examination. The patient recovered cyclosporine and mycophenolate mofetil on the first day after operation and refused to accept postoperative adjuvant chemotherapy. Peritoneal and paraaortic lymph nodes were discovered recurrence 12 months after operation and died due to tumor progression 3 months later. This suggests that we should monitor the occurrence of gastrointestinal tumors after liver transplantation and intervene early to obtain a higher survival rate. Chemotherapy should also be used as adjuvant treatment when necessary.

RETRACTED

Due to the risk of radioactive liver disease, the application of external beam radiotherapy in the treatment of hepatocellular carcinoma is limited. Other treatment options for advanced liver cancer include systemic chemotherapy, chemoembolization, radiofrequency ablation, percutaneous ethanol injection, and radioembolization. Radioembolization with 90Y glass microspheres is particularly useful for patients with advanced HCC who are not suitable for resection [68].

### 3.8. Adjuvant Therapy

The selection of postoperative adjuvant therapy is related to the type of new tumor, the degree of malignancy, and the location of transplanted organs. Systemic chemotherapy or radiotherapy is usually limited to advanced cases and recurrent diseases [69].

The standard treatment of head and neck squamous cell carcinoma (HNSCC) includes initial surgery in the early stage of the tumor, followed by adjuvant radiotherapy (RT)/chemoradiotherapy (CRT) or initial CRT alone in patients with advanced HNSCC [26]. However, considering the results of this high-risk patient population, there is no evidence-based recommendation for the optimal treatment of patients with new HNSCC after liver transplantation.

Prostate cancer after renal transplantation is the second common malignant tumor of the urinary system. The treatment methods are radical prostatectomy, external beam radiotherapy, and androgen deprivation. The choice of treatment was based on age, comorbidity, and Gleason score. Patients undergoing surgery were younger. Patients receiving radiotherapy, with a total dose of 76 Gy, irradiated the prostate and excluded the upper pelvic area to protect the graft from potential radiation injury. Patients receiving androgen deprivation therapy died of causes unrelated to cancer several months later [70].

The treatment of PTLD after transplantation depends on its subtype. Early type and polymorphic PTLD usually respond to reduced immunosuppression and rituximab monotherapy, while monomorphic PTLD usually requires additional concurrent or sequential chemotherapy. For rare subtypes of PTLD, standard of care guidelines for neonatal lymphoma are recommended. According to the degree of disease, surgical resection or radiotherapy can be used as adjuvant treatment. Nonchemotherapy such as adoptive T cell therapy has shown promising efficacy and must be further studied [71].

RETRACTED

Although the site of concurrent malignancy is usually not in the same area as the transplanted organ, the outlining of the radiotherapy target area is still an important step in precision radiotherapy; however, there are not many studies reported empirically on the adjustment of radiation dose.

### 3.9. Palliative Care

In the cases of de novo esophageal tumors after liver transplantation reported by Presser et al. [68], the corresponding treatment plan was formulated according to the patient's physical condition. A total of 5 patients (50%) received conservative treatment. The definite radiotherapy and chemotherapy included 60 Gy irradiation and cisplatin-based chemotherapy. If the esophagus is so narrow that the patient cannot eat, the patient can repeatedly receive palliative expansion or laser coagulation. The other 5 patients were generally in good condition and underwent radical lymph node dissection to achieve the purpose of treatment.

In addition, transcatheter arterial chemoembolization has also been widely used in palliative treatment of patients with large tumors, but its survival benefit is uncertain [72].

## 4. Discussion

Cancer, recurrence of primary diseases, cardiovascular disease, and infection are the four most common causes of long-term death after transplantation [73]. The tumors of liver transplant recipients can be divided into four types: (1) donor transmission cancer (DTC), that is, it exists in allografts at the time of transplantation; (2) donor-derived carcinoma (DDC), which develops in donor cells after transplantation; (3) new cancer, as a long-term result of transplantation, develops from recipient cells; (4) recurrent cancer refers to the recurrence of cancer treated before transplantation and after transplantation [74].

The development of cancer is a multifactorial process. The effective immune system recognizes and attempts to eliminate primary tumors via cytotoxic T lymphocytes, macrophages, and natural killer cells, which can recognize tumor cells as nonself cells (so-called immune surveillance), delay tumor progression, and prevent angiogenesis, vascular infiltration, and metastasis [75]. The immune system can also control virus infection with carcinogenic ability, but in transplant recipients, immunosuppressive drugs destroy immune function by promoting cell transformation and escaping immune recognition and directly affect the site of tumor formation [76]. The transmission of malignant tumors by donors, long-term exposure to risk factors or potential carcinogens, the growth of age, smoking, and drinking may be the inducing factors of tumors [77]. According to single factor analysis reported by Desai and Neuberger [74], age, gender, Caucasian, past malignancies, multiple organ transplantation, alcoholic liver disease, primary sclerosing cholangitis, and nonalcoholic steatohepatitis were associated with primary diseases, obesity, diabetes, age of donors, and use of mTOR inhibitors during transplantation. Donor factors (age, gender, race, and obesity) and recipient creatinine are not risk factors for malignant tumors after liver transplantation. Some studies have also shown that the survival rate after concurrent tumors is related to gender. Women could better survive after being diagnosed with malignant tumors, which is not suitable for patients with skin cancer or lymphoma [78]. The author believes that the cause of posttransplant malignant tumor is the use of immunosuppressants, which leads to systematic immunosuppression and the recipients are more vulnerable to pathogen invasion. In the meantime, the human body can not produce enough antibodies to resist the invasion of antigen, so that the cancer cells is possible to proliferate continuously. Another reason is that the body is in the state of immunosuppression for long so that the original normal flora in the body becomes pathogenic bacteria leading to carcinoma.

RETRACTED

According to the morbidity of malignant tumor after organ transplantation, the data of different countries and centers are different. According to the data screened in this review, the incidence of malignant tumors after organ transplantation is 0.2%~22.8%. According to the results of our review, the morbidity of malignancies after liver transplantation is relatively high. The author believes that the reasons for the high risk of tumors after liver transplantation may be related to the spread of malignant tumors by donors and the unhealthy habits like smoking and drinking by recipients. Patients who have to undergo liver transplantation usually have the habit of smoking and drinking or carry hepatitis virus, coupled with bad living habits, which are easy to induce cancer. The morbidity of skin cancer in European countries is relatively high after operation, which may be related to skin color, sunshine radiation, and immunosuppressive agents. The incidence rate of gastrointestinal cancer is higher in Korean and Japanese patients. In China, the incidence rate of urologic tumor is high, and the mechanism may be related to, which is Chinese patent medicine containing aristolochic acid [79].

The treatment of malignant tumors is generally based on surgery. Radical cancer resection can remove tumors, reduce tumor metastasis, and prolong the survival of patients. However, the patient is usually so late to found when the tumor was usually advanced and metastasized, that operation could not be performed. Patients who have no tumor metastasis and are suitable for surgery can be treated surgically [37]. The effect of the surgery is related to the type, size, and stage of the tumor; physical conditions such as there are other concurrent diseases and whether to choose the chemotherapy may also infect the survival of the patient, but there are few relevant articles. The specific treatment methods should be selected by clinicians according to the patient's condition.

RETRACTED

The choice of postoperative adjuvant therapy should be based on the patient's age, the degree of malignancy of the tumor. For patients after organ transplantation, we had better monitor the tumor regularly, intervene in the early stage, and give adjuvant radiotherapy and chemotherapy when physical conditions permit.

A study on different forms of diagnosis and treatment of esophageal cancer patients without organ transplantation showed that patients who underwent surgical resection after neoadjuvant radiotherapy and chemotherapy had a higher survival rate than those who received radiotherapy and chemotherapy alone. The five-year survival rate of patients with radiotherapy and chemotherapy or radiotherapy alone is only 6~27%, but the five-year survival rate of patients with surgical resection after radiotherapy and chemotherapy can reach 17~49% [68].

Tacrolimus is the most common choice of immunosuppressants, and standard immune triple therapy is wildly used in clinic. However, because tacrolimus has the risk of causing cancer, it is now clinically recommended to minimize CNI or replace CNI with mTOR inhibitors, which plays the role of chemical prevention and protect renal function. Rapamycin also has a good effect on Kaposi's sarcoma. Therefore, clinicians need to decide the medication according to the specific situation of patients.

According to the current diagnosis and treatment, patients with tumors after organ transplantation should continue to take immunosuppressants. CNI can be minimized or mTOR inhibitors can be used to replace CNI. The choice of postoperative adjuvant therapy should be based on the type and spread of cancer and personal physical conditions. When the tumor is relatively limited, radiotherapy can be selected, and its side effects are relatively small. When the tumor diffusion degree is relatively high, chemotherapy should be selected to inhibit cancer cells in the whole body.

In a word, there is no clear standard in the diagnosis and treatment of this kind of patient with malignant tumors after organ transplantation. The current diagnosis and treatment method is to maintain immunosuppression and add adjuvant treatment such as surgery or radiotherapy and chemotherapy. However, there is no in-depth study on the effect of antitumor drugs on transplanted organs. The existing research results can provide limited guidance for clinical practice, and we look forward to more optimized and clear treatment strategies which bring more benefits to patients with malignant tumors after organ transplantation.

RETRACTED

We have compiled and analyzed the development and treatment of malignancies complicating organ transplantation and summarized the treatment recommendations based on the available studies. Due to the small number of organ transplantation cases and the lack of research and data on antitumor treatment options, there are limitations in our analysis, such as the lack of research data on targeted therapy and immunotherapy, which prevents us from giving treatment recommendations for such patients. However, as the number of organ transplantation cases continues to increase, research data in this area will continue to increase and we will need to keep an eye on the treatment of this patient population.

## Figures and Tables

**Figure 1:** Tumor morbidity of postrenal transplant recipients.

**Figure 2:** Tumor morbidity of postliver transplant recipients.

**Table 1:** Types of carcinoma in postrenal transplant patients.

Author	Year	Region	Patient in total	DNM	Renal	Gastrointestinal	Other urological cancers	Respiratory cancer	Female reproductive system	PTLD and blood *t*	Skin and Kaposi	Head and neck	Prostate	Breast	Others	Time of tumor diagnosis (Y)
Fröhlich et al. [9]	1995-2016	UK	1417	154	49	30	24	18	15	14	NA	NA	NA	NA	29	5.8
Park et al. [15]	2007-2015	North Korea	10085	289	58	100	13	36	17	52	45	4	14	30	72	2.9
Gioco [13]	2000-2012	Italy	535	39	5	3	1	6	NA	2	9	NA	1	2	10	3
Mazzucotelli et al. [10]	1997-2012	Italy	735	75	11	7	2	5	NA	26	12	NA	12	7	NA	1.7
Rossetto et al. [12]	1995-2010	Italy	636	59	11	17	4	3	2	NA	3	1	2	3	18	NA
Wu et al. [16]	1989-2010	China	1467	14	3	1	7	1	NA	1	NA	NA	NA	NA	2	3.6
Apel [8]	1966-2005	German	1882	231	22	43	16	14	19	7	NA	NA	5	NA	12	2.8
Tsai et al. [7]	2003-2009	Taiwan, China	186	35	NA	8	19	1	NA	4	1	NA	NA	0	1	NA
Zavos et al. [11]	1983-2013	Turkey	2054	199	5	23	2	14	9	26	99	NA	6	6	9	8
Sampaio et al. [14]	1999-2008	USA	123380	4179	431	540	158	637	93	892	55	NA	446	307	115	2.8

Note: NA: not mentioned; Y: year.

**Table 2:** Types of carcinoma in postliver transplant patients.

Author	Year	Region	Patients in total	DNM	Renal	Gastrointestinal	Other urological cancers	Respiratory cancer	Female reproductive system	PTLD and blood *t*	Skin and Kaposi	Head and neck	Prostate	Breast	Others	Time of tumor diagnosis (Y)
Egeli et al. [20]	1998-2016	Turkey	429	9	NA	NA	NA	5	NA	NA	1	2	NA	NA	1	5.3
Park et al. [15]	2007-2015	South Korea	3822	213	4	100	2	13	7	35	11	6	NA	9	26	1.9/3.0^c^
Hegab et al. [21]	2001-2010	Saudi Arabia	238	8	NA	NA	1	NA	1	5	1	NA	NA	NA	NA	3.6
Ettorre et al. [22]	1990-2008	Italy	1675	98	NA	18	6	25	NA	22	6	19	NA	3	7	3.2
Carenco et al. [23]	1991-2008	France	465	106	NA	15	8^a^	15	NA	13	31	17	8^∗^	4	3	6.3 ± 4.3^d^
Rademacher et al. [24]	1988-2006	German	1616	266	19^∗^	51	19^b^	59	11	NA	83	NA	9	19	15	8.1^e^
Sanaei et al. [25]	1992-2012	Turkey	1700	38	NA	6	NA	NA	NA	24	3	NA	NA	NA	5	5.6
Mizuno et al. [26]	2002-2017	Japan	97	11	NA	3	1	1	NA	4	1	1	NA	NA	NA	8.3
Sampaio et al. [14]	1999-2008	USA	43106	1923	37	457	277	386	26	456	12	45	155	85	7	2.6

a: including both prostate and urogenital tumors; b: including both renal and urogenital tumors; c: 1.9 years for hematopoietic cancer, 3 years for patients with nonhematopoietic cancers; d: for solid organ cancers; e: 8.1 for solid organ tumors; NA: not mentioned; Y: year.

RETRACTED

## Data Availability

The datasets used and/or analyzed during the current study are available from the corresponding author on reasonable request.
